The article "Detection of Pancreatic Cancer in CT Scan Images Using PSO SVM and Image Processing" was retracted in 2024. Reasons: signs of a paper mill; suspected computer-generated content; unreliable results or conclusions; concerns about the data.

# Detection of Pancreatic Cancer in CT Scan Images Using PSO SVM and Image Processing

**DOI:** 10.1155/2022/8544337

**Published:** 2022-07-26

**Authors:** Arshiya S. Ansari, Abu Sarwar Zamani, Mohammad Sajid Mohammadi, Meenakshi, Mahyudin Ritonga, Syed Sohail Ahmed, Devabalan Pounraj, Karthikeyan Kaliyaperumal

**Affiliations:** ^1^Department of Information Technology, College of Computer and Information Sciences, Majmaah University, Al-Majmaah 11952, Saudi Arabia; ^2^Department of Computer and Self Development, Preparatory Year Deanship, Prince Sattam Bin Abdulaziz University, Al-Kharj, Saudi Arabia; ^3^Department of Information Technology, College of Computer, Qassim University, Buraydah, Saudi Arabia; ^4^GD Goenka University Sohna Haryana, India; ^5^Universitas Muhammadiyah Sumatera Barat, Indonesia; ^6^Department of Computer Engineering, Qassim University, Buraydah, Saudi Arabia; ^7^BVC Engineering College (Autonomous), Odalarevu, Allavaram Mandal, East-GodhavariDistrict, Andhra Pradesh, India; ^8^IT @ IoT-HH Campus, Ambo University, Ethiopia

## Abstract

A diagnosis of pancreatic cancer is one of the worst cancers that may be received anywhere in the world; the five-year survival rate is very less. The majority of cases of this condition may be traced back to pancreatic cancer. Due to medical image scans, a significant number of cancer patients are able to identify abnormalities at an earlier stage. The expensive cost of the necessary gear and infrastructure makes it difficult to disseminate the technology, putting it out of the reach of a lot of people. This article presents detection of pancreatic cancer in CT scan images using machine PSO SVM and image processing. The Gaussian elimination filter is utilized during the image preprocessing stage of the removal of noise from images. The *K* means algorithm uses a partitioning technique to separate the image into its component parts. The process of identifying objects in an image and determining the regions of interest is aided by image segmentation. The PCA method is used to extract important information from digital photographs. PSO SVM, naive Bayes, and AdaBoost are the algorithms that are used to perform the classification. Accuracy, sensitivity, and specificity of the PSO SVM algorithm are better.

## 1. Introduction

A diagnosis of pancreatic cancer is one of the worst cancers that may be received anywhere in the world; the five-year survival rate is only 9.3 percent. The majority of cases of this condition may be traced back to pancreatic cancer (American Cancer Society, 2017). One of these organs is the pancreas, which is the organ that comes after the liver in the digestive system. There are a few species of fish that have heads, bodies, and tails that are all deceptively similar to one another in appearance. Even after it is grown to adult size, the width is just around 5 centimeters (about 2 inches) [1, 2].

The article "Detection of Pancreatic Cancer in CT Scan Images Using PSO SVM and Image Processing" was retracted in 2024. Reasons: signs of a paper mill; suspected computer-generated content; unreliable results or conclusions; concerns about the data.

It is possible for a condition known as pancreatic adenocarcinoma to develop when exocrine cells in the pancreas grow in an uncontrolled manner. This particular form of pancreatic cancer occurs the most frequently. Exocrine cells are what make up the ducts and glands that are known as exocrine organs. These organs are located in the pancreas and are responsible for the secretion of fluid. These glands, which are known as exocrine glands and can be found in the digestive tract, are responsible for the production of enzymes that are of assistance in the digestion of food [3].

The pancreatic duct is the ultimate resting place for enzymes after they have been secreted into ducts, which are very thin tubes. The bile that is produced by the liver is expelled into the ampulla of the Vater during the digestive process. This occurs after the bile has passed through the regular bile conduit. The pancreatic duct eventually makes its way into the ordinary bile conduit and joins it there. Endocrine cells, which are a smaller percentage of the cells that make up the organ but produce essential hormones such as insulin and glucagon, which regulate and release blood sugar levels directly into the circulation, are the cells in the pancreas that are responsible for the development of the pancreatic tumor. These cells are responsible for the growth of the pancreatic tumor [4], despite the fact that they make up a lesser percentage of the cells that make up the organ.

Even though the vast majority of pancreatic growths are benign, which means they do not cause cancer, there are some of them that have the potential to develop into cancer if they are not treated. These growths are known as precancers. Imaging tools like as magnetic resonance imaging (MRI), computed tomography (CT), ultrasound, positron emission tomography (PET), and positron emission tomography combined with computed tomography (PET/CT) scans are helpful in the detection of certain pancreatic [5]. One image showing pancreatic cancer is shown in Figure 1

Since image processing and computer modelling are the most common techniques used in medical imaging, biomedical imaging has attracted a diverse variety of imaging technologies. Researchers of biological and microbiological data still rely heavily on the participation of humans in a huge majority of their studies. Inherent in physical processes are the human propensity for biased interpretations of those processes, the unpredictability that exists among human specialists, as well as lengthy and expensive procedures. In order to carry out an analysis that is both objective and recursive, accurate quantitative measurements, the examination of huge datasets, and the use of technologies that are automated are necessary [6, 7].

The article "Detection of Pancreatic Cancer in CT Scan Images Using PSO SVM and Image Processing" was retracted in 2024. Reasons: signs of a paper mill; suspected computer-generated content; unreliable results or conclusions; concerns about the data.

There is also the possibility for cancer burden reduction to be achieved through early detection and treatment options. If many cancerous growths are found at an early stage and given appropriate treatment, there is a good possibility that all of them can be eliminated. It is necessary for the World Health Organization (WHO) to make an effort in order to close the discovery gap in this situation and progress the process of early identification of cancerous development. Recent changes and upgrades have been made to the infrastructure of the research facilities. The development and widespread use of novel approaches to the early detection of cancer are now underway. The identification of people who seek medical attention for cancer-related symptoms and are ultimately given a cancer diagnosis has been the focus of recent efforts. On the other hand, a significant number of people who have cancer go undiagnosed or are only diagnosed and treated after significant delays.

Due to medical image scans, a significant number of cancer patients are able to identify abnormalities at an earlier stage. The expensive cost of the necessary gear and infrastructure makes it difficult to disseminate the technology, putting it out of the reach of a lot of people. As a result, heavy-duty radiography of expert quality and in-depth analysis are not readily available. Because of this, and concerns about the low accuracy of image-based cancer diagnosis as well as significant intra- and interreader variability, earlier WHO guidelines for resource-limited settings emphasized that medical scan pictures should be used primarily when cancer is not proven with lab tests and biopsies. This recommendation was made in light of the fact that medical scan pictures should be used [8].

Radiologists rely on computer-aided diagnostic tools to assist them in interpreting the images of patients' medical conditions. Using image processing and machine learning algorithms applied to CT scans, it is possible to identify pancreatic cancer at an earlier stage.

Literature survey contains a review of existing work in the field of pancreatic cancer detection and classification. Methodology contains proposed methodology. The Gaussian elimination filter is utilized during the image preprocessing stage of the removal of noise from images. The *K*-means algorithm uses a partitioning technique to separate the image into its component parts. The process of identifying objects in an image and determining the regions of interest is aided by image segmentation. The PCA method is used to extract important information from digital photographs. PSO SVM, naive Bayes, and AdaBoost are the algorithms that are used to perform the classification. Result Analysis contains experimental results. Accuracy, sensitivity, and specificity of PSO SVM algorithm are better.

The article "Detection of Pancreatic Cancer in CT Scan Images Using PSO SVM and Image Processing" was retracted in 2024. Reasons: signs of a paper mill; suspected computer-generated content; unreliable results or conclusions; concerns about the data.

### 1.1. Literature Survey

Suhas and Venugopal [9] employed a technique that included median and mean filtering in order to remove noise from medical images. This strategy was part of their overall approach. It has been suggested that an innovative technique be used that makes use of linear as well as nonlinear filters. The median and mean filter values are utilized in order to obtain a more accurate reading of each pixel in an image that contains noise. A comparison was made between the recommended method and filters based on the mean, the median, and the halfway using numerical metrics such as PSNR, SNR, and RMSE. The results of this comparison were compared to the typical pattern of sounds. It has been proved that the structural details of a medical picture may be kept when using this technology, while at the same time, the image noise can be significantly decreased. When using this experimental method, MRI photos will have a higher degree of precision.

Denoising medical images required the application of the median and Wiener filters, as stated in Anitha et al. [10]. The median filter is a type of image filter that, like the mean filter, is used to reduce the amount of noise in a picture. However, unlike the mean filter, the median filter does so without affecting the image's fine details. When the median filter is applied to a specific pixel, an intensity level will have its value changed to be the median of the other neighboring intensity levels. Pixels that have had their quality reduced might always be substituted for those that are considered to be good. The amount of noise that the Wiener filter eliminates from an audio stream is determined by first doing an analysis of what the sound of a signal that is free of noise should be like. The only method to ascertain the answer is through the use of statistical analysis. In order to arrive at this conclusion, the pixel size and clarity of a picture are assessed and compared to a conventional noise pattern. In terms of filtering and overall performance, the median filter was the clear winner over the other filters. Photos filtered using the median have a higher pixel quality than images filtered with the Wiener filter.

Lakshmi and colleagues [11] have developed a preprocessing method that is based on soft computing techniques for the purpose of functional MRI data segmentation. Image denoising that is based on the curvelet transform is a very effective method for getting rid of noise. Quantitative testing will need to be increased since further clinical scans and realistic phantoms are going to be required in order to validate the method's precision and consistency.

The article "Detection of Pancreatic Cancer in CT Scan Images Using PSO SVM and Image Processing" was retracted in 2024. Reasons: signs of a paper mill; suspected computer-generated content; unreliable results or conclusions; concerns about the data.

An improvement has been made to a technique that was created by Rong and Yong [12] in order to remove salt and pepper noise from an image. Visual noise is identified using Median Filter 2.0, which then generates a noise-marked matrix that takes into consideration the characteristics of the found noise. In this particular instance, the processing skips over the pixel that has been determined to be a signal. On the other hand, the median filter is the one that is used the most frequently since it has a fantastic ability to get rid of background noise and a wonderful efficiency when it comes to computing. The task of the median filter is to replace the grey value of each pixel with the median value of its neighbors. When there is a significant quantity of noise, image features become obscured. The author came up with an improved method for median filtering by making use of local histograms. This method is able to keep the image's finer details intact. The histogram is utilized to determine which noise pixels have a significant amount of impulsivity. The histogram provides a visual representation of the number of noise detections that occurred for each conceivable value of the grey scale in pixels. A significant increase in the peak value of the histogram provides irrefutable evidence of the presence of impulse noise. The performance of enhanced median filters has been examined by subjecting them to testing with various noise densities ranging from 10% to 50% with an increase of 10% in each step. These performance metrics demonstrate that the technique that was advised is more effective in cutting down on background noise. According to the findings of the experiment, not only does it a better job of preserving the picture's details but it is also more suited for the routine de-noising of images on computers.

In this particular study, it was Gao and colleagues [13] that investigated the segmentation of 4D CT scans for nodules (taken at different points in time). It has been recommended that this criterion, which takes into account the degree to which the images of the different phases are similar to one another, be added into the graph cut approach in order to reduce the size of the energy function. This strategy has the downside of requiring manual segmentation to be performed in the very beginning of the process.

The article "Detection of Pancreatic Cancer in CT Scan Images Using PSO SVM and Image Processing" was retracted in 2024. Reasons: signs of a paper mill; suspected computer-generated content; unreliable results or conclusions; concerns about the data.

Ju et al. came up with a different strategy that is based on the graph cut [14]. This approach, which takes use of the data obtained from CT and PET imaging, can have its accuracy improved by the application of cosegmentation. This approach uses a random walk algorithm in order to generate the starting seeds for the graph cut technique. Graph cut is a technique for cutting graphs. This strategy makes use of two subgraphs: one for PET pictures and one for CT images. Both of these subgraphs are connected to one another via a particular connection that penalizes the difference in segmentation that results from using the two different modalities. The next step in lowering the energy function is to increase the flow while simultaneously minimizing the cuts.

In the hybrid cost function that Mukherjee and his colleagues created, deep learning and domain-specific knowledge are integrated [15]. The second set of authors proposes a strategy that begins with graph cut segmentation and then concludes with CNN. The use of convolutional neural networks (CNN) as a filter to eliminate false positives is at the heart of this methodology.

Lee and colleagues [16] developed a color image segmentation algorithm that is based on particle swarm optimization and takes saliency into consideration (PSO). When computing the saliency map, spatiotemporal feature maps are put to use. This map is then put to use to guide the area merging process, which is carried out with a modified PSO and an image segmentation hybrid fitness function for color.

Akila and Sumathy [17] proposed an innovative method for the segmentation of color images by combining local histogram equalization (LHE) with *K*-means clustering. LHE is a method for enhancing color photographs that works by changing pixels and making use of the information contained inside the image. In the end, a color picture is segmented by the use of the *K*-means clustering approach. After that, this method is contrasted with some other tried-and-true approaches, such as the subtractive clustering, fuzzy *C*-means, and *K*-means approaches.

The paper [18] devised a method for segmenting medical images using principal component analysis (PCA) and *K*-means clustering. This method isolates the areas of the image that are most pertinent to the study. *K*-means is the process of clustering is one method that may be utilized to single out significant aspects of an image. Increasing the use of principal component analysis (PCA) in the process of feature extraction and determining the optimal number of clusters is one way to enhance accuracy. A novel approach was developed in order to increase the reliability of illness diagnosis through the use of MRI image segmentation.

The article "Detection of Pancreatic Cancer in CT Scan Images Using PSO SVM and Image Processing" was retracted in 2024. Reasons: signs of a paper mill; suspected computer-generated content; unreliable results or conclusions; concerns about the data.

Surlakar conducted a quick comparison of the segmentation techniques of *K*-means and *K*-nearest neighbor in the field of medicine [19]. These algorithms have been tested using cells derived from tumors. It has been demonstrated that the *K*-nearest neighbor approach is more effective in the process of picture segmentation based on mutual assessment criteria. The *K*-means approach produced satisfactory segmentation outcomes for *k* values that were lower than 1. The segmentation, on the other hand, gets progressively coarse as *k* increases, which results in a scattering of clusters over the images.

An ANN-based image classifier was utilized by Arunkumar and Murthi [20] for the purpose of performing early identification of pancreatic tumors. The fact that an abdominal ultrasound does not offer information on the stage of the tumor and does not capture the microscopic tumors that are picked up by an MRI or CT scan is a significant disadvantage. They utilized a neural network-based image classifier in order to increase the percentage of patients who make a full recovery and detect pancreatic tumors at an earlier stage utilizing PET scan images.

Using an artificial neural network model that Olufemi and his colleagues created, it is feasible to diagnose pancreatic cancer. The Levenberg-Marquardt back propagation technique was utilized throughout the training process of the network. Utilizing this approach, we were able to diagnose pancreatic cancer at a variety of stages. The results demonstrated an accuracy rate of 87 percent, which demonstrates the advantages of utilizing an ANN model [21].

Only MRI photos are capable of identifying the tumorous region due to image processing, which employs *K*-means segmentation and image preprocessing. Adaptive brain tumor detection was proposed by Swapnil et al. [22]. In order to make this system more flexible, an unsupervised SVM (support vector machine) was used to build and store the pattern for later application. This was done to make the system more versatile. Finding a feature that can be used to train SVM on is an issue that patterns face as well. Because of this, they have conducted an analysis of the area's texture as well as its color. It is anticipated that the results of the experiments conducted using the proposed system would be superior to those conducted using competing systems.

A comparison was made between the modified self-organizing map (SOM) network and the conventional SOM network for the purpose of medical picture analysis [23]. During the analysis of the dataset, thirty ultrasound photographs of the breast, ten images of the brain obtained from an MRI scan, and one image of the skull obtained from a CT scan were seen. The input feature space of the network is built with the help of a DWT, which stands for discrete wavelet transform. The filtering features of the network contribute in many different ways to the reduction of visual noise. The Jaccard index, the Rogers index, and the Tanimoto index all agree that the strategy that has been recommended provides more accurate results than the SOM-based network method.

The article "Detection of Pancreatic Cancer in CT Scan Images Using PSO SVM and Image Processing" was retracted in 2024. Reasons: signs of a paper mill; suspected computer-generated content; unreliable results or conclusions; concerns about the data.

Hashem and his colleagues [24] came up with several ideas automating the classification of mammograms, and they presented those ideas. First, the image is described with the help of feature extraction techniques, and then, it is categorized with the assistance of machine learning algorithms. Texture descriptors from the first and second orders of statistics were utilized in order to provide an analysis of mammography images. A decision tree (DT), a random forest (RF), a naive Bayes (NB) algorithm, a C4.5 algorithm, and a multilayer perceptron (MLP) algorithm were employed to identify the pictures (DT). Their ultimate goal is to determine the optimal combination of feature extraction and classification algorithms that will result in precise mammogram classifications. This will allow them to achieve their target. It was determined that the most successful method for classifying mammography images was to use a mix of second-order statistics and random forest.

The accuracy of a machine learning algorithm's cancer prediction is dependent on the data collection and the characteristics of the data [25]. There are a variety of methods that are utilized to classify data, including support vector machines, random forests, naive Bayes, decision trees, *K*-nearest neighbors, artificial neural networks, fuzzy neural networks, RBFN, shuffled frog leaping with levy flights, particle swarm optimization, back propagation neural networks, multilayered perceptron, and SVM recursive feature elimination. According to the findings of this research, the support vector machine (SVM) method of machine learning is the most effective method for predicting cancer sickness from a given dataset.

### 1.2. Methodology

This section presents detection of pancreatic cancer in CT scan images using machine PSO SVM and image processing. To remove noise from images, image preprocessing is performed by Gaussian elimination filter. Image is partitioned in to segments by *K*-means algorithm. Image segmentation helps in object identification and deciding region of interest. Relevant features from images are extracted using PCA algorithm. Classification is performed by PSO SVM, naïve Bayes, and AdaBoost algorithm. This is shown below in Figure 2.

The article "Detection of Pancreatic Cancer in CT Scan Images Using PSO SVM and Image Processing" was retracted in 2024. Reasons: signs of a paper mill; suspected computer-generated content; unreliable results or conclusions; concerns about the data.

There are several different morphological activities that may be taken to lessen or eliminate background noise. The median filtering technique may be used to adjust the brightness of the pixels, while the Gaussian filtering technique can be used to smooth out the images. Both techniques can be combined. In this particular instance, the Gaussian filter was used to achieve noise reduction (GF). The properties of the picture are preserved by the application of a weighted average of the intensities of neighboring pixels; nevertheless, the importance of the intensity at each pixel is changed. Using this technology, it is feasible to smooth photos while maintaining the borders of the images. Smoothing is done to the picture using Gaussian kernels by applying accumulative standard deviation [26].

*K*-means clustering is a kind of pattern that divides the many interpretations into *k* different clusters, each of which is connected to a different cluster that has the local mean. The approach makes advantage of the total number of groups that are represented by *k* in order to locate groups within a dataset. It determines the closest data points by using squared Euclidean distances in its calculations. In accordance with the characteristics that were selected, each data point was put into one of the *k* different categories. The data points are categorized according to how closely their characteristics align with one another [27].

The approach known as principal component analysis (PCA) is used to carry out the process of feature extraction. It is possible that the linear technique of principal component analysis (PCA) to dimensionality reduction may be helpful in the process of data analysis and compression [28]. It is possible to combine a large number of uncorrelated characteristics by using this strategy, which involves finding orthogonal linear combinations of the characteristics that were originally included in the dataset.

For nonprobabilistic binary linear classification, the best method is the particle swarm optimization support vector machine. “Particle swarm optimization” is what “PSO-SVM” stands for as an acronym. Because of its ease of use and broad applicability, the PSO (particle swarm optimization) method has been effectively used in the cancer classification process. This method allows for the separation of samples into a single target class as well as into a large number of target classes. Every bit of information is represented by a single point in this chart. It continues to become broader as a result of the significant distinctions that exist between each successive group. Depending on which side of the gap new instances land on, the target classes of newly created instances may be remapped. It is feasible to do nonlinear classification when the datasets being inputted are not labelled. In order to classify the data, the support vector machine makes use of an unsupervised learning strategy. This is necessary due to the fact that the instances cannot be assigned to target classes. After the formation of the clusters based on functions, further instances are added to the database. Evidence suggests that a nonlinear support vector machine recommendation system is in operation. When it comes to dealing with unlabeled data, the nonlinear support vector machine technique is the one that is used most often [29].

The article "Detection of Pancreatic Cancer in CT Scan Images Using PSO SVM and Image Processing" was retracted in 2024. Reasons: signs of a paper mill; suspected computer-generated content; unreliable results or conclusions; concerns about the data.

Bayes' theorem provides the foundation for the Bayesian classification system and serves as its basis. These naive Bayesian classification techniques, when applied to a large database, are able to characterize simple bases in a manner that is analogous to the classification of end trees and selected networks. The naive Bayes classification is able to represent a restricted number of dependent qualities because to this feature. Using this technique, an estimate can be made for the probability *P* (*x*|*c*) for each class. The classes that were found in this research to have the greatest probability served as the basis for the prediction of the results [30].

(1) $$\begin{array}{c} P\left(c\left|x\right.\right)=\frac{P\left(x\left|c\right.\right)\;P\left(c\right)}{P\left(x\right)}, \end{array}$$

where the *P*(*c*|*x*) posterior probability of each class given diabetes x attribute, *P*(*x*|*c*) is the likelihood value, *P*(*c*) is the prior probability of diabetes class, and *P* (*x*) is the prior probability of predictor.

Each attribute conditionally forgives the subset class.

In AdaBoost decision tree, a different base classification has a weighted dataset if the weight of a single instance in the dataset depends on the previous base classifier results for each of these instances [31]. If they misunderstand an instance, the weight of that instance will increase in future models, and if the classification is correct, the weight will remain the same [31].

### 1.3. Result Analysis

The medical segmentation decathlon (MSD) dataset [32] has 420 abdomen CT scans of patients with different pancreatic tumors. 280 images were used for training and remaining 140 images are used for testing of model. To remove noise from images, image preprocessing is performed by Gaussian elimination filter. Image is partitioned in to segments by *K*-means algorithm. Image segmentation helps in object identification and deciding region of interest. Relevant features from images are extracted using PCA algorithm. Classification is performed by PSO SVM, naïve Bayes, and AdaBoost algorithm. Three parameters accuracy, sensitivity, and specificity are used in this study to compare performance of different algorithms. Accuracy, sensitivity, and specificity of PSO-SVM, naïve Bayes, and AdaBoost classifiers for pancreatic cancer tissue detection are shown below in Figure 3.

(2) $$\begin{array}{c} \text{Accuracy}=\frac{\text{TP}+\text{TN}}{\left(\text{TP}+\text{TN}+\text{FP}+\text{FN}\right)}, \end{array}$$

(3) $$\begin{array}{c} \text{Sensitivity}=\frac{\text{TP}}{\text{TP}+\text{FN}}, \end{array}$$

(4) $$\begin{array}{c} \text{Specificity}=\frac{\text{TN}}{\text{TN}+\text{FP}}, \end{array}$$

where TP indicates true positive, TN indicates true negative, FP indicates false positive, and FN indicates false negative.

The article "Detection of Pancreatic Cancer in CT Scan Images Using PSO SVM and Image Processing" was retracted in 2024. Reasons: signs of a paper mill; suspected computer-generated content; unreliable results or conclusions; concerns about the data.

## 2. Conclusion

It is one of the worst diseases that may be diagnosed anywhere in the world; the five-year survival rate is quite low. Pancreatic cancer is one of the worst tumors that can be diagnosed. One of the most common causes of this syndrome is pancreatic cancer, which accounts for the majority of cases. A sizeable percentage of cancer patients are now able to detect anomalies at earlier stages because to the increased availability of medical imaging scans. It is difficult to propagate the technology because of the high cost of the necessary gear and infrastructure, which puts it out of reach for a significant number of people. This article discusses the use of machine PSO SVM and image processing for the purpose of detecting pancreatic cancer in CT scan pictures. The CLAHE method is applied during image preprocessing in order to clean up photos that have noise. The *K*-means method uses a partitioning technique to separate the image into its component parts. The process of identifying objects in an image and determining the regions of interest is aided by image segmentation. The PCA method is used to extract important information from digital photographs. PSO SVM, AdaBoost, and C4.5 are the algorithms that are utilized for the classification process.

## Figures and Tables

**Figure 1:** CT scan image of pancreatic cancer tissue.

**Figure 2:** Detection of pancreatic cancer in CT scan images using machine PSO SVM and image processing.

**Figure 3:** Result comparison of machine learning for pancreatic cancer detection.

## Data Availability

The data shall be made available on request.
